RETRACTED

# Effect of Annular External Fixator-Assisted Bone Transport on Clinical Healing, Pain Stress and Joint Function of Traumatic Massive Bone Defect of Tibia

**DOI:** 10.1155/2022/9052770

**Published:** 2022-07-15

**Authors:** Xiaoliang Song, Xinzhong Shao

**Affiliations:** ^1^Hand Surgery, The Third Hospital of Hebei Medical University, Shijiazhuang, Hebei 050000, China; ^2^Department of Orthopaedics, Changzhi Second People's Hospital, Changzhi, Shanxi 046000, China

## Abstract

**Objective:**

To investigate the effect of annular external fixator-assisted bone transport in the treatment of traumatic massive bone defect of tibia on clinical healing, pain stress, and joint function.

**Methods:**

From January 2018 to November 2021, 146 patients with traumatic massive bone defect of tibia were selected as the research objects, and they were divided into observation group (annular external fixator-assisted bone transport, 71 cases) and control group (unilateral external fixator bone lengthening, 75 cases) according to different surgical methods. The therapeutic efficacy, fracture healing-related indexes, and postoperative range of motion of the knee joint were compared between the two groups. Callus healing was evaluated by Fernandez-Esteve callus score, and joint function was evaluated by Paley score, American Knee society score (AKSS), and Baird-Jackson ankle score. The changes of pain mediator (serum substance P (SP), neuropeptide Y (NPY), prostaglandin E2 (PGE2), and tumor necrosis factor-*α* (TNF-*α*)) and stress indexes (adrenocorticotropic hormone (ACTH), cortisol (COR), and nor Epinephrine (NE)) were observed before and after treatment in two groups. The incidence of postoperative complications was analyzed.

**Results:**

There were no significant differences in total effective rate and bone lengthening between the two groups (*P* > 0.05). The bone healing time and callus formation time in the observation group were shorter than those in the control group, and the Fernandez-Esteve callus score was higher than that in the control group (*P* < 0.05). The levels of SP, NPY, PGE2, TNF-*α*, ACTH, COR, and NE in the observation group were lower than those in the control group (*P* < 0.05). AKSS and Baird-Jackson scores in the observation group after operation were higher than those in the control group (*P* < 0.05). There was no significant difference in the incidence of postoperative complications between the two groups (*P* > 0.05).

**Conclusion:**

Annular external fixator-assisted bone transport can promote postoperative fracture healing, reduce pain stress level, and improve joint function of patients with traumatic massive bone defect of tibia.

RETRACTED

## 1. Introduction

Acute bone injury, infection, and nonunion can all cause traumatic bone defects, which account for about 0.4% of all fractures. The lack of soft tissue coverage on the anteromedial aspect of the tibia makes traumatic bone defects the most common (68% of all bone defects) due to high-energy injury [1]. Tibial fractures caused by high-energy trauma or open tibial fractures with secondary infection often leads to bone and soft tissue defects after debridement, especially massive bone defects, which seriously affect the clinical treatment and prognosis of patients [2, 3]. Bone transport is a major treatment for massive bone defect of tibia, and some studies have pointed out that bone transport can effectively improve the surgical efficacy [4]. The main technical principle is to transport the bone segment adjacent to the defect area to the bone defect area by osteotomy technique. During the transport process, with the action of distraction osteogenesis, new bone will be generated in the osteotomy area so that the bone segment can be healed with the contralateral bone end [5]. At present, there are two kinds of external fixation systems commonly used in bone transport: unilateral external fixator and annular external fixator. According to previous literature, unilateral external fixator bone lengthening is one of the effective methods for the treatment of traumatic massive bone defect of tibia. It can repair bone defects of any length without bone grafting, and the ossification rate of new bone callus is faster, which can greatly shorten the bone healing time, and the operation method is relatively simple compared with the annular external fixator [6, 7]. However, this method still has some limitations, and some patients still have no improvement in knee and ankle function after treatment [8]. In addition to the advantages of unilateral external fixator, the annular external fixator has higher stability and can help patients get out of bed early [9]. Although the curative effect of the annular external fixator-assisted bone transport for the treatment of massive bone defect of tibia is clear, there is no clear report on the effect of this surgical treatment on the release of pain mediators and postoperative stress level of patients. Therefore, the purpose of this study was to investigate the effects of annular external fixator-assisted bone transport on clinical healing, pain stress, and joint function of traumatic massive bone defect of tibia and to provide clinical reference for the treatment of this disease.

## 2. Materials and Methods

### 2.1. Clinical Data

From January 2018 to November 2021, 146 patients with traumatic massive bone defect of tibia were selected as the study subjects. According to different surgical methods, they were divided into observation group (annular external fixator-assisted bone transport, 71 cases) and control group (unilateral external fixator-assisted bone lengthening, 75 cases). The inclusion criteria are as follows: (1) Patients who met the diagnostic criteria for large tibial bone defect: X-ray examination showed that the length of the tibial bone defect was more than 5 cm [10]; (2) all patients with tibial fractures were caused by accidents; (3) patients with clinical indications for the treatment of large tibial bone defect by transplantation [11]: The degree of bone defect must exceed 5cm; the bone shape was long tubular, and the distal and proximal ends can be fixed with stents; no acute infection; bone on one side of the bone; the body length was longer to allow bone transport; and the limbs were intact; (4) the patients had informed consent and signed the informed consent; (5) age ≥ 18 years old; (6) those with complete clinical data; and (7) patients with high compliance. Exclusion criteria are as follows: (1) patients with contraindications related to surgical treatment; (2) patients with old fractures; (3) patients with osteoporosis; (4) patients with a history of tibial surgery; (5) patients with severe blood system diseases; (6) patients complicated with severe organ dysfunction; (7) patients with severe diabetes; and (8) patients with fractures at other sites.

RETRACTED

### 2.2. Methods

Patients in the control group were treated with unilateral external fixator-assisted bone lengthening. After anesthesia, the patient was placed in supine position and fixed with a unilateral external fixator. The operation area was carefully treated, the lesions and surrounding necrotic tissue were completely removed, the wound surface and the bone marrow cavity of the residual bone were washed repeatedly, and the bone defect of the lesion site was examined by X-ray. The knee joint of the affected limb was slightly flexed, from the fibulae capitulum, passed through the tibia in internal-frontal direction; the needle was inserted backward by crossing the anterior needle at a 60° angle through the lateral side of the medial anterior piercing point and, in the same way, inserted through the upper side of the lateral malleolus to the position at 4 cm from the ankle joint surface. During the osteotomy, an incision of about 2 cm was made on both sides of the anterior tibial crest, and the long periosteum was cut lengthwise. The nerve stripper was used for circumferential dissection to maintain the integrity of the periosteum. The affected limb was raised; bone lengthening and regular X-ray review were performed after operation, extending 0.1-0.2 cm per day, divided into three times. X-ray films were taken at 2, 4, 6, and 8 weeks after the operation to observe the recovery. Routine anti-infection, improvement of microcirculation, and anti-inflammatory symptomatic treatment were applied postoperatively. Functional activities of adjacent joints were performed 2 days after operation, and the surrounding skin was kept clean and dry during the wear of extension frame. Stitches were removed 2 weeks after the operation.

RETRACTED

The observation group was treated with annular external fixator-assisted bone transport, and the patients were given basic symptomatic treatment such as debridement and hemostasis after admission. After anesthesia, the patient was placed in supine position and fixed with an annular external fixator. After adjusting the corresponding fixator according to the limb length of the patient's unaffected side, the corresponding Kirschner wire was inserted into the ring at the distal and proximal ends of the tibia of the affected limb to facilitate the installation of the external fixator. At the same time, the corresponding Kirschner wire was inserted into the bone body, and the annular external fixator was installed to maintain the force line of the affected limb and the length of the tibial fracture end. Small incisions were made at the corresponding distal and proximal ends of the tibia, the metaphysis was stripped annularly, and the corresponding osteotomy was performed under the periosteum. Patients with simple skin lesions were treated with negative pressure suction, and patients with skin defects and bone exposure were treated with gastrocnemius muscle flap. Routine anti-infection, improvement of microcirculation, and anti-inflammatory symptomatic treatment were also applied postoperatively. Functional activities of adjacent joints were performed 2 days after operation. Bone transport was performed 1 to 2 weeks after the fixation, and X-ray films were also taken at 2, 4, 6, and 8 weeks after the operation to observe the recovery. The lengthening speed was adjusted according to the ratio of the minimum diameter of callus and the diameter of osteotomy end suggested by the examination results, and the compression was carried out after the contact between the two broken ends was ensured. In addition, X-ray reading adopted double review of the image results. If there was any objection, please ask a senior third person to verify and judge to ensure the accuracy and reliability of the results.

### 2.3. Observation Indicators

#### 2.3.1. Clinical efficacy

Clinical efficacy of patients was evaluated according to Paley grading [12], which was divided into 4 grades: excellent, good, general, and poor. Excellent: fracture healing, no recurrent infection, local deformity angle less than 7°, unequal length of limb less than 2.5 cm, no obvious claudication, slight joint stiffness, angle of knee extension or ankle dorsiflexion decreased by less than 15° compared to that before operation, and no reflex sympathetic dystrophy; good: fracture healing, no recurrent infection, local deformity angle less than 7°, obvious claudication, reflex sympathetic dystrophy, and obvious pain; general: fracture healing, no recurrent infection, able to complete normal daily activities, obvious claudication and reflex sympathetic dystrophy; and poor: fracture nonunion, recurrent infection, local malformation angel greater than 7°, obvious claudication, reflex sympathetic dystrophy, and obvious pain.

RETRACTED

#### 2.3.2. Fracture Healing–Related Indicators

Bone lengthening length and bone healing time were compared between the two groups.

#### 2.3.3. Callus Healing

The callus formation time and the Fernandez-Esteve callus score were compared between the two groups [13], and the Fernandez-Esteve callus scoring method was used to evaluate the callus healing of the patients, and the score ranged from 0 to 4 points. 0 points indicated no radioactive callus at the fracture end, 1 point indicated cloudy callus at the fracture end, 2 points indicated the presence of one side callus on the frontal and lateral view of the fracture end, 3 points indicated the presence of bilateral callus on the frontal and lateral view of the fracture end, and 4 points indicated the presence of structural callus formation.

#### 2.3.4. Pain Mediators

3 ml of fasting venous blood was collected 1 day before surgery and 3 days after surgery, and the serum was separated by centrifugation. Serum substance P (SP), neuropeptide Y (Neuropeptide Y, NPY), prostaglandin E2 (PGE2), and tumor necrosis factor-*α* (TNF-*α*) were detected by Hitachi 7200 automatic biochemical reaction analyzer and supporting reagents.

#### 2.3.5. Stress Response

Adrenocorticotrophic hormone (ACTH), cortisol (COR), and norepinephrine (NE) were detected 1 day before surgery and 3 days after surgery by enzyme-linked immunosorbent assay.

#### 2.3.6. Joint Function

Baird-Jackson ankle joint score was used to evaluate the ankle joint function of patients 1 day before operation and 3 months after operation [14], mainly including 7 aspects such as pain, ankle stability, walking ability, running ability, and working ability. The score ranges from 0 to 100 points, and the higher the score, the better the recovery of joint function. The American Knee Society Score (AKSS) was used to evaluate the knee joint of patients 1 day before surgery and 3 months after surgery [15], which was divided into knee score and functional score. The knee score is divided into pain, range of motion, and stability, and the functional score includes the ability to walk and go up and down stairs. Each score ranges from 0 to 100 points, and the higher the score, the better the knee function. The scoring index adopts single-blind tests and double scoring and takes the average score.

RETRACTED

### 2.4. Statistical Processing

SPSS22.0 software was used to process data, count data was expressed as percentage, and *χ*^2^ test was used to compare differences between groups; measurement data were expressed as ^−^x ± s after normality test, and *t* test was used to compare differences between groups. *P* < 0.05 indicated that the difference was statistically significant.

## 3. Results

### 3.1. Comparison of the General Data of the Two Groups of Patients

There was no significant difference in the general data of the two groups of patients (*P* > 0.05), as shown in Table 1.

### 3.2. Comparison of Therapeutic Effects between the Two Groups

There was no significant difference in the total effective rate of surgery between the two groups (*P* > 0.05), as shown in Table 2.

### 3.3. Fracture Healing–Related Indicators between the Two Groups

There was no significant difference in the length of bone lengthening between the two groups (*P* > 0.05). The bone healing time and callus formation time in the observation group were shorter than those in the control group, and the Fernandez-Esteve callus score was higher than that in the control group (*P* < 0.05), as shown in Figure 1.

### 3.4. Comparison of Postoperative Pain Mediator Levels between the Two Groups

There was no significant difference in the levels of SP, NPY, and PGE2 between the two groups before surgery (*P* > 0.05); the levels of SP, NPY, and PGE2 in the observation group 3 days after surgery were lower than those in the control group (*P* < 0.05), as shown in Figure 2.

### 3.5. Comparison of Stress Indicators between the Two Groups

There was no significant difference in the preoperative stress indicators between the two groups (*P* > 0.05); the levels of TNF-*α*, ACTH, COR, and NE in the observation group 3 days after operation were lower than those in the control group (*P* < 0.05), as shown in Figure 3.

### 3.6. Comparison of AKSS and Baird-Jackson Scores between the Two Groups

There was no significant difference in the preoperative AKSS and Baird-Jackson scores between the two groups (*P* > 0.05). The postoperative AKSS and Baird-Jackson scores of the observation group were higher than those of the control group (*P* < 0.05), as shown in Figure 4.

RETRACTED

### 3.7. Comparison of the Incidence of Complications between the Two Groups

There was no significant difference in the incidence of postoperative complications between the two groups (*P* > 0.05).

## 4. Discussion

Tibia is a kind of subcutaneous bone vulnerable to trauma, and its fracture is mostly open, which is more common in long bone fracture. Clinically, the massive bone defect of tibia is mostly caused by high-energy injury, and patients are often accompanied by serious tissue injury of muscles, nerves, and blood vessels [16, 17]. Bone transport technique is a common method for the treatment of traumatic massive bone defect of tibia, and it can achieve a good therapeutic effect. However, unilateral external fixator treatment has poor stability and high risk, which can affect the treatment effect and lead to poor prognosis of patients, for example, it is not conducive for patients to get out of bed early for activities and functional exercise, and the recovery of joint function is slow [18–20]. In addition, the traction needle of unilateral external fixator is thick, which stimulates bone and soft tissue greatly and is easy to be infected. However, the annular external fixator-assisted bone transport for the treatment of traumatic massive bone defect of tibia can effectively avoid the inflammatory area caused by the bone defect, and the external fixator can effectively prevent the further spread of infection through the form of needle threading structure [21]. In this study, the effective rate of this method was as high as 90.14%, indicating the high clinical efficacy of annular external fixation-assisted bone transport in the treatment of traumatic massive bone defect of tibia. The reason may be that during the treatment in this study, bone transport was performed within 2 weeks after the operation, which could effectively ensure that the normal blood supply and circulation of the bone tissue of the skin flap and the recipient skin had been restored, and would not cause unnecessary influence on the blood supply of the skin flap during the bone transport, which can promote the healing of broken bone ends and the repair of soft tissue, which is beneficial to the recovery of patients [22]. In addition, this study found that the time of bone healing and callus formation in the observation group was shorter than that in the control group and Fernandez-Esteve callus score was higher than that in the control group, suggesting that annular external fixator-assisted bone transport for the treatment of traumatic massive bone defect of tibia can promote callus formation and bone healing. This study believes that this is also an important factor for the high surgical efficacy of this operation.

RETRACTED

SP is a kind of neuropeptide distributed in the thin primary afferent nerve fibers, which can directly or indirectly promote the release of glutamate and other substances, and participate in the process of pain transmission; NPY is a polypeptide secreted by hypothalamus, which is widely distributed in central and peripheral nervous system and plays an indicative role in pain stress; PGE2 is an important cell generation and regulatory factor, which is closely related to the process of pain stress [23, 24]. Surgical trauma is an important factor affecting postoperative pain, and the release of pain mediators is closely related to the degree of pain. Relevant reports indicate that the release of pain mediators is related to wound size and surgical site [25]. It has also been reported that acute trauma is in a state of high stress; due to the release of pain-causing and inflammatory mediators, it can not only aggravate the ischemia, hypoxia, and edema of the primary lesion, but also cause abnormal metabolism of hormones and enzymes in the body, which can affect the prognosis of patients in serious cases [26]. In this study, the levels of SP, NPY, and PGE2 in the observation group decreased 3 days after surgery, indicating that the use of annular external fixator-assisted bone transport for the treatment of traumatic massive bone defect of tibia can effectively inhibit the release of pain mediators, and thus may play a role in alleviating postoperative pain. However, the specific mechanism is still unknown, so further analysis is needed in the later stage to explore the effect of this operation on pain mediators. In addition, TNF-*α* is a potent proinflammatory cytokine, which involved in the acute phase stress response [27]. The main function of ACTH is to promote the secretion of cortisol by the adrenal cortex to maintain the normal physiological function and metabolism of the human body, and ACTH and COR were elevated in the human body under stress [28]. In a state of stress, the secretion of NE increases rapidly, causing the following changes in the body: increased heart rate, increased blood pressure, increased physical fitness, and increased vigilance [29]. In this study, the postoperative levels of TNF-*α*, ACTH, COR, and NE in the observation group were lower than those in the control group, indicating that the postoperative stress level of the body can be reduced by the annular external fixator-assisted bone transport for patients with traumatic massive bone defect of tibia. The reason is that the surgical operation space is small and the influence on the internal environment of the body is small during this operation, which is beneficial to reduce postoperative inflammatory response and stress level [30].

RETRACTED

The tibia is the bone that supports the inner side of the human lower leg, and it plays an important role in normal walking and exercise. Traumatic massive bone defect of tibia can cause the loss of the function of the weight-bearing lower leg and affect the joint function. Clinical data show that the treatment of massive bone defect of tibia is different from simple fracture, which only needs to be fixed and healed, and the treatment of bone defect needs to repair the patient's bone and limb morphology [31]. The external fixator can effectively avoid further damage to the soft tissue of the fracture site during the treatment of bone transport, and there is no need to strip the periosteum during the operation, thus ensuring the blood supply to the tibial fracture end, and thus improving the joint function. In addition, during bone transport, the location of the osteotomy is selected at the epiphysis, where the blood supply is relatively abundant, which can contribute to fracture healing and improve the postoperative motor ability and quality of life of patients [32]. The results of this study showed that the AKSS and Baird-Jackson scores in the observation group were higher than those in the control group, suggesting that annular external fixator-assisted bone transport can improve the function of knee joint and ankle joint in patients with traumatic massive bone defect of tibia. This is mainly because this surgical treatment can effectively ensure the healing of the grafted bone, and the limb can not only achieve bone lengthening, but also complete the extension of skin and other soft tissues under the effect of tensile stress, which plays a positive role in promoting the balance of lower limb movement and wound repair [33, 34]. In addition, the traction needle used in annular external fixator is thinner, which has less stimulation to bone and soft tissue less susceptible to infection and less painful. In this study, there was no significant difference in the incidence of postoperative complications between the two groups, indicating that this surgical treatment is relatively safe. However, patients in the annular external fixator group had lower pain levels and better recovery of limb function after surgery.

In conclusion, annular external fixator-assisted bone transport for the treatment of traumatic massive bone defect of tibia can promote postoperative fracture healing, reduce the level of pain and stress, and improve the joint function of patients. There are still some shortcomings in this study. The included patients in this study are few, and the observation time is short, which may affect the final results. And the pain and stress indicators were only studied 1 day before surgery and 3 days after surgery, but the start time of bone transfer was different between the observation group and the control group, so more observations should be set time point for comparison. Therefore, it is necessary to increase the sample size and prolong the observation time in the later stage to further explore the effect of this operation on the prognosis of patients.

RETRACTED

## Figures and Tables

**Figure 1:** Fracture healing-related indicators between the two groups.

**Figure 2:** Comparison of postoperative pain mediators between the two groups.

**Figure 3:** Comparison of stress indicators between the two groups.

**Figure 4:** Comparison of AKSS and Baird-Jackson scores between the two groups.

**Table 1:** Comparison of general data of the two groups of patients.

Item	Observation group (*n* = 71)	Control group (*n* = 75)	*χ* ^2^/*t*	*P*
Age (years)	43.05 ± 7.13	44.29 ± 7.52	1.021	0.309
Gender (male/female)	44/27	41/34	0.800	0.371
Bone injury length(cm)	7.92 ± 1.26	8.05 ± 1.18	0.644	0.521
Cause of injury (cases)			0.375	0.829
Traffic accident injuries	34	37		
High falling injury	21	19		
Collision by heavy objects	16	19		
Injured site (cases)			0.5021	0.479
Middle end of the tibia	42	40		
Middle and lower end of the tibia	29	35		

**Table 2:** Comparison of therapeutic efficacy between the two groups (cases, %).

Group	*n*	Excellent	Good	General	Poor	Excellent and good rate
Observation group	71	28	36	4	3	90.14
Control group	75	27	32	9	7	78.67
*χ* ^2^						3.618
*P*						0.057

## Data Availability

The labeled dataset used to support the findings of this study are available from the corresponding author upon request.
